The article "An Annealing Model Analysis and Research on the In of Community Public Sports on Economic Development" was retracted in 2023. Reasons: unreliable results or conclusions; concerns about the data; concerns about the results or conclusions; concerns about the peer review.

# An Annealing Model Analysis and Research on the In of Community Public Sports on Economic Development

**DOI:** 10.1155/2022/3129638

**Published:** 2022-04-15

**Authors:** Zhen Guo

**Affiliations:** School of Physical Education, Shaoyang University, Shaoyang 422000, China

## Abstract

The state vigorously develops the application of community sports and takes it as an important unit of social and economic development. With the development of the economy, residents' living standards are getting better, which also greatly promotes the development of community public sports. Community public sports have made great progress in terms of scale, hardware, and services, and their impact on society is getting worse. Come bigger. However, there are still some deficiencies in the development of community sports. How to accurately evaluate and predict its facilities, construction, and service levels and put forward corresponding development strategies is an urgent problem to be solved in the field of community public sports. In this paper, an iterative simulated annealing algorithm is proposed to evaluate the level of public sports services and help community public sports institutions identify their own development deficiencies. Through the simulation analysis of the community sports organizations, community members, venue facilities and funds, venue facilities and funds, administrators, and the community sports activities, it is found that the identification accuracy of the evaluation results of the five indicators is above 95%, while the initial threshold of community public sports and social and economic development and the prediction accuracy required by the standard of development status are both 10%. At the same time, the recognition time of the evaluation results in the five indicators is less than 7 seconds. In community public sports development trend prediction and service level judgment, the identification time of the evaluation result is less than 4 seconds, and the overall judgment result is better.

## 1. Introduction

With the development of digitization and computers, public sports and other related industries have developed rapidly, showing the characteristics of rapidity, diversity, and intelligence shown by Sadegh Barkhordari and Tehranizadeh [1]. Community sports mainly refer to the regional mass sports carried out nearby in a certain area where people live together, taking the natural environment and sports facilities of the jurisdiction as the material basis, taking all community members as the main body, and taking meeting the sports needs of community members, increasing the physical and mental health of community members, and consolidating and developing community feelings as the main purpose. Community sports have six elements: community sports organizations, community members, venues, facilities and funds, administrators, instructors, and community sports activities. Public sports are affected by external and internal factors and cannot be accurately evaluated and analyzed by traditional data analysis methods, which affects the evaluation effect of service level (Bourliva et al. [2]) and limits the development of intelligent public sports. Some scholars believe that the purpose of the intelligent development of community public sports is to meet the development needs of the industry. Therefore, starting from the prediction of development trend, operation status, and the development of community public sports (Donoso [3]), a comprehensive evaluation of the public sports service level can provide a reference for the formulation of a service strategy. Some scholars also believe that the accuracy of intelligent evaluation in community public sports is low, and the proportion of unstructured data is high (Durmus [4]).

We can improve the accuracy of intelligent evaluation of public sports and reduce the interference of unstructured data by extracting eigenvalues. Based on the above background, this paper uses metropolis acceptance criteria and a simulated annealing algorithm to analyze the eigenvalues and analyzes the service level of community public sports from the perspective of intelligence so as to improve the evaluation accuracy of public sports services. Based on the above reasons, this paper mainly introduces it from three aspects. Firstly, it describes the service level in the community of public sports mathematically, and introduces the intelligence of service level, the parameters of service level, and the processing of service level-related data. Secondly, a prediction model of public sports service level based on a simulated annealing algorithm is constructed. The constraints of the simulated annealing algorithm, the accuracy of public sports service level, and the prediction steps of public sports service level are analyzed. Thirdly, the simulation of public sports service level prediction model is based on a simulated annealing algorithm. We describe the cases of public sports services and analyze the accuracy and calculation time of prediction results.

From the above analysis, it can be seen that the rapid development of community public sports can promote the development of the social economy and make its decision-making develop in a positive direction. In order to better carry out the research of community public sports and make them play a role in economic promotion, it is necessary to introduce comprehensive judgment methods to improve the accuracy of calculation, which is of great practical significance. In addition, the comprehensive analysis of community public sports can also enhance the coupling between community public sports and economic development and provide support for development decision-making.

## 2. The Mathematical Description of Service Level Prediction in Community, Public Sports, and Social Economy under Simulated Annealing Algorithm

The iterative simulated annealing algorithm is a comprehensive calculation method, which can carry out iterative analysis on community public sports. This algorithm has the advantages of a simple calculation process and fast analysis speed. Compared with the classical simulated annealing algorithm, the iterative simulated annealing algorithm can carry out progressive calculation, eliminate redundant data, make the calculation result more accurate, and avoid local extremum.

### 2.1. The Intelligent Description of Service Level

Intelligent service level has two characteristics: on the one hand, it processes massive information, uncertain data, and diverse data, and the proportion of controllable data is >50%; on the other hand, multisource data are analyzed and dynamic information is obtained. The public sports data structure is as follows: the diversity of data sources, the comprehensiveness of public sports, and the diversity of calculation, observation, and measurement (Fitriningsih [5]), as shown in Figure 1.

The structure of public sports data is mainly in the form of controllable and uncontrollable factors and is combined with the economic data sources of public sports-related industries to form a large amount of public sports data. Public sports should start from the industry, conduct intelligent analysis in combination with industry development capacity, industry service status and trend, and improve the accuracy of public sports assessment.

It can be seen from Figure 2 that although the demand for sports for community public sports fluctuates, it is increasing on the whole. Therefore, community public sports play a vital role in the development of sports. Some scholars also believe that community public sports can also promote the development of a social economy. The specific contents are shown in Figure 3.

It can be seen from Figure 3 that there is a certain correlation between social public sports and the social economy, and the correlation is increasing year by year. In summary, community-based public sports play a supportive role in sport development and are somewhat correlated with social and economic development. In order to better carry out the development of community public sports and give play to their social promoting role, it is necessary to conduct in-depth research on community public sports. At the same time, depending on the current situation of public community sport, foresee its future development, in order to improve the development of sport and the social economy. As a result, a thorough analysis of community public sports is of great practical and theoretical importance.

### 2.2. Description of Service Level Metrics

The digitization of the level of public sports services and the diversification of the factors influencing demand increasingly highlight the characteristics of public sports data. The traditional level of service method cannot fully address the intelligent development needs of community-based public sports. Under the background of intelligent development, public sports prediction algorithms such as particle swarm optimization and support vector can meet the needs of large volume and multiple types and realize the prediction and analysis of public sports service level, community public sports service status, and public sports development trend. The parameters of the community public sports are set as follows (Haghverdi [6]): community sports organizations, community members, venue facilities and funds, administrators, directors, and coordinators of community sports activities.

(1) Assume the community sports organizations are *x_i_*, the community members are *x_j_*, community outdoor fitness venues and funding are *x_k_*, venue facilities and funds are *x_l_*, administrators are *x_m_*, the community sports activities is *x_n_*, and the intelligent dataset of the community public sports service level is C. The result of the calculation shall be drawn up in accordance with the following formula:
  (1) $$\begin{array}{c} C=\left\{c_{1},c_{2},\ldots \ldots c_{i}\right\}, \end{array}$$
where *c*_*i*_ is shown in the following formula:
  (2) $$\begin{array}{c} c_{i}=\bar{\sum_{i,j,k}^{n}x_{i}+x_{j}+x_{k}+x_{l}+x_{m}+x_{n}}, \end{array}$$
where *I*,  *j*,  *k*,  *l*,  *m*,  *n* belongs to natural numbers. The different data for the public service of sport come from different sectors.
(2) Suppose *n* is an intelligent collection, *i* is the industry of data source, *j* is the structure type of data (uncontrollable factor data = 1, otherwise = 0), *k* is the data acquisition method (qualitative method acquisition = 1, quantitative method acquisition = 2, comprehensive acquisition method = 0), *l* is the intelligent development level (Note: 1∼5 levels, the higher the value, the higher the level), and *M* is each data collection organization, then the data acquisition item can be described as *N*_*i,j,k,l,M*_,*i*, *j*, *k*, *l*, *M* = (1, 2,…, *n*), and *n* is a natural number.
(3) Different public sports institutions divide similar industry sources, structure types, acquisition methods, and economic development level data into community public sports data sets.
(4) Data from all data institutions are analyzed centrally by the Centre for Economic Analysis of Community Public Sport. Under the constraints of forecast accuracy, prediction time, and safety, the data obtained are classified according to the relevant weights and thresholds.
(5) The collection time of health data and the intelligence level of health data in any given data organization are the same or similar (Han [7]).
(6) For the stability of the data organization and analysis, the Fourier series method shall be adopted to reduce the interference of data organization, personnel, and other nonresistance factors as shown in the following formula:
  (3) $$\begin{array}{c} P\left(t\right)=a_{0}+\sum_{\text{i}=1}^{n}\frac{\left[\left(y_{i}z_{i}u_{i}-y_{i-1}z_{i-1}u_{i-1}\right)\right]}{2}+\frac{\left(y_{i}z_{i}u_{i}+y_{i-1}z_{i-1}u_{i-1}\right)}{2}+\xi , \end{array}$$
where *P* is the antiinterference ability described by the intelligent analysis of health data, i*t* is the measured time of health data, wh*y* is the degree of intelligence, *z* is the interval of health data collection, yo*u* are the sports health standard, and *ξ* interference coefficient.

### 2.3. Simplified Processing of Health Information Data

The data gathered by the various public sports institutions must first be processed by K-means. The result is indicated in the form equation as follows:

(4) $$\begin{array}{c} \sum_{i=0}^{n}I_{i}=\left|S\right|. \end{array}$$

Among them, *S* is the clustering range, the lower the value, the better the clustering effect. *I* is the data collected by the data organization, and *I* is the number of the data. In addition, *S* can be replaced by similarity *J* so as to improve the efficiency of the calculation. In order to simplify the process, the weight can be judged by using the frequency of a certain date, the data threshold collected by the data institution can be judged according to the previous historical data or the data frequency in the community public sports database, that is shown in the following formula:

(5) $$\begin{array}{c} w_{i}=\frac{H\cdot G_{ij}}{G_{i}+G_{j}}, \end{array}$$

where *G*_*ij*_ is the number of times *J* data organization collects *I* data, *G*_*i*_ is the number of times *I* data appears in the community public sports database, *G*_*j*_ is the frequency *j* data organization sends data, and *WI*_*i*_*s* the threshold of *my* data.

## 3. Construct a Public Sport Intelligence Prediction Model Based on a Simulated Annealing Algorithm

### 3.1. The Limitations of the Simulated Annealing Algorithm

Prior to the analysis of intersectoral data institutions in the community, public sports, all data institutions should be classified and judged according to applicable standards. In this paper, the metropolis acceptance criteria (Harkut et al. [8]) are adopted. If community-based public sports meet real needs, relevant data will be collected, otherwise, data organizing data will not be accepted. Metropolis accepts the judgment of the criteria and can save the resources of the community public sports, reduce the amount of data processing, and improve the speed of intelligent development (Luo et al. [9]). Assuming that the state of the community public sports is *the*, we conduct metropolis acceptance criteria analysis to determine whether the state needs to be changed, that is, from *my* state to *i* + 1 intelligence. The calculation formula shall be

(6) $$\begin{array}{c} R\left(T\right)\left\{\begin{array}{c} R\left(T\right)=0∼0.5,\\ R\left(T\right)=0.5∼1. \end{array}\right) \end{array}$$

The limitations of formula (2) appear in formula (7)as follows:

(7) $$\begin{array}{c} \left\{\begin{array}{c} f\left(i\right)⟶f\left(i\right),\\ f\left(i+1\right)⟶f\left(i+1\right),\\ \text{exp}\left[\frac{f\left(i\right)-f\left(i+1\right)}{T_{i}}\right], \end{array}\right) \end{array}$$

where exp() is the expected function of service intelligence, which is to judge whether to be smart; *R*(*T*) is the result function of intelligence in community public sports. If the result of *R*(*T*) is 0∼0.5, it indicates that the degree of intelligence is low and the original state can be maintained. If the result ranges from 0.5 to 1.

### 3.2. The Appropriateness between Collective Sports and the Recut Algorithm

The adjustment of communal public sports and the annealing algorithm is divided into (Luo [10]) local adjustment CP and global adjustment MP, which reflect the adjustment of the two under different aspects, which is also the premise of the calculation of the evaluation results. The larger the values of *PC* and *Pm*, the better the data fit. Since metropolis in 2.1 accepts the limitation of the criterion and requires both data to be optimized in order to become the calculation data, the calculation formula is as follows:

(8) $$\begin{array}{c} P_{\text{c}}\left(\begin{array}{cc} N_{1,1,0,1}, & R_{c}=R_{mg},\\ \frac{\varphi_{c}\left(R_{c}-R_{\min}\right)}{\left(R_{mg}-R_{\min}\right)}, & R_{c}<R_{mg}, \end{array}\right.. \end{array}$$

(9) $$\begin{array}{c} P_{\text{m}}\left(\begin{array}{cc} N_{1,1,1,0}, & R_{m}=R_{mg},\\ \frac{\varphi_{m}\left(R_{m}-R_{\min}\right)}{\left(R_{m}-R_{\min}\right)}, & R_{m}<R_{mg}, \end{array}\right.. \end{array}$$

where *N*_1,1,0,1_ is the initial value of *P*_c_, *N*_1,1,1,0_ is the initial value of *P*_m_, *R*_min_ is the minimum value of the whole data, *R*_*c*_ is the local minimum value, and *R*_*m*_ is the overall minimum value. *φ*_*c*_ is the local fitting coefficient and *φ*_*m*_ is the overall fitting coefficient.

### 3.3. The Accuracy of the Results for Predicting the Level of Public Sport Intelligence

The corresponding datasets should be constructed before the prediction results are calculated. In this paper, the appropriate function is used to clarify the relationship between the simulated annealing algorithm and community public sports (Martin-Fernandez [11]). Under the conditions of preset accuracy and threshold constraints, the moderate function performs multiple iterative analyses, guides the operator to calculate in the positive direction, reduces the occurrence rate of local extreme values and “false eigenvalues” (Petroff [12]), and improves the accuracy of predictive results, as shown by the following formula:

(10) $$\begin{array}{c} f\left(x⟶y\right)=\min\left[\int_{i,j}^{n}\sum_{i=1}^{n}\max\left(F\left(x_{i}\right),F\left(x_{i+1}\right)\right),\sum_{j=1}^{n}\max\left(y_{j}\right),\left(y_{j+1}\right)\right]+{∲}_{i}\sin\left(\xi_{i}\right), \end{array}$$

where *f*(*x*⟶*y*) is the relationship function between simulated annealing algorithm and community public sports, that is, the appropriate function, which reflects the matching degree between them. The maximum value of any two service data is as follows:

(11) $$\begin{array}{c} \sum_{i=1}^{n}\max\left(F\left(x_{i}\right),F\left(x_{i+1}\right)\right). \end{array}$$

The maximum value expected from any level of intelligence is as follows:

(12) $$\begin{array}{c} \sum_{j=1}^{n}\max\left(y_{j}\right),\left(y_{j+1}\right). \end{array}$$

The level of information provided by public sports institutions to obtain the maximum or minimum of two points is as follows:

(13) $$\begin{array}{c} \int_{i,j}^{n}\left(\sum_{i=1}^{n}\max\left(F\left(x_{i}\right),F\left(x_{i+1}\right),\sum_{j=1}^{n}\max\left(y_{j}\right),\left(y_{j+1}\right)\right)\right). \end{array}$$

The minimum of all extreme values is set out as follows:

(14) $$\begin{array}{c} \min\left[\int_{i,j}^{n}\sum_{i=1}^{n}\max\left(F\left(x_{i}\right),F\left(x_{i+1}\right)\right),\sum_{j=1}^{n}\max\left(y_{j}\right),\left(y_{j+1}\right)\right]. \end{array}$$

### 3.4. Steps in Predicting Community Public Sports Based on a Simulated Annealing Algorithm

Using the above mathematical description, the following calculations are needed:

1. We set initial *C* = {*c*_1_, *c*_2_,…, *c*_*i*_} values of community public sports, thresholds of data fitting (local fitting *Pc*, overall fitting *Pm*) and calculation accuracy, intelligent prediction results *N*_*i*_, *j*, *k*, *l*, _*m*_ values, and initial metropolis acceptance criteria;
2. Gradient 200 iterative tests were performed on the fitted data (Reinaldi [13]);
3. We verify the calculation results according to metropolis acceptance criteria and constraints, incorporate the qualified results into the total scheme, and calculate the recognition accuracy and calculation time of the prediction results of the overall scheme (Ren e al. [14]);
4. We determine whether all the data we are going through will stop the calculation, otherwise proceed to step 3;
5. Finally, the minimum value should be taken out. The overall diagram and output of the computation process are shown. The specific process is presented in Figure 4.

## 4. Case Analysis of the Public Sports Information Prediction Model Based on a Simulated Annealing Algorithm

### 4.1. The Case Introduction

We take 4 provincial public sports establishments, 5 municipal public sports establishments, and 6 county public sports establishments from January 1, 2020, to December 2021 as examples. Song et al. [15] analyze the impact of the simulated annealing algorithm on the current state and trend of development of public sports services and determine the accuracy of the discrimination and time of the prediction results. The accuracy and calculation accuracy of data fitting (partial fitting PC and overall fitting PM) are set to 0.1 and the number of iterations is 200. Among them, the data collection is the statistical yearbook of public sports institutions, the website of public sports institutions, and a questionnaire survey (reliability and validity >0.7). The intelligence level is level 3 and follows the guidelines for the development status of community public sports (GB/T 31464) in 2015, The IP addresses of public sports institutions are 192.168.1.102∼192.168.1.202.

### 4.2. The Fit between Community Public Sports and Simulated Annealing Algorithm

Through K-mean clustering and metropolis acceptance criteria, the data of intelligent and public sports industries are standardized, and 20 iterative analyzes are carried out to obtain the data fitting results, as shown in Table 1.

It can be seen from Table 1 that both local fitting and overall fitting are >95%, while the overall fitting is high and meets the threshold of 10% set by K-mean clustering and metropolis acceptance criteria. The results of the specific couplings are presented in Figure 5.

It can be seen from Figure 6 that there is a strong correlation between community public sports and social economy, which shows that community public sports present a large-scale and high-level development trend and can promote economic development and make it develop in a positive direction. At the same time, the rapid development of the economy also promotes the upgrading and development of community sports. For the classical simulated annealing algorithm, the iterative simulated annealing algorithm has a higher correlation, indicating that the correlation between social public sports and economic development is stronger, which lays the foundation for accurate calculation in the later stages.

### 4.3. Community Public Sports and the Social Economy

The results show that although the correlation between social public sport and social economy fluctuates in a small range, the overall correlation is high, between–20% and 180%. As a result, there is a strong relationship between community public sports and the social economy. The small fluctuation between community public sports and social economy is mainly determined by the whole society's sports policy and social-economic policy, and has nothing to do with the simulation results of the annealing algorithm in this paper. The specific outcomes are presented in Figure 6.

### 4.4. The Accuracy of Prediction Results

The community sports organizations are *x*_*i*_, the community members are *x*_*j*_, the venue facilities and funds are *x*_*k*_, the venue facilities and funds are *x*_*l*_, the administrators are *x*_*m*_, and the community sports activities are *x*_*n*_. The accuracy of the identification of predictive results in the five indicators directly determines the effectiveness of the entire model.

Through MATLAB simulation analysis, it can be seen that the recognition accuracy of the prediction results in the abovementioned five indicators is >95%, while the initial threshold and the requirements in the criteria for the current service situation of community public sports are 0.1. At the same time, in the process of 40∼50 iterations, the calculation accuracy changes greatly, which is mainly caused by the jumping change in social and economic development and does not affect the final calculation accuracy. So, the simulation results are better, and the results are shown in Table 2.

The precision of the specific calculation can be derived from the data in Table 2, and the results are illustrated in Figures 7–9.

It can be seen from Figure 8 that the service judgment result of social public sports is better, which is between 75 and 99% as a whole, better than 82∼89% of the classical simulated annealing algorithm. We can see that the computation result of the iterative simulation annealing algorithm is better.

It can be seen from Figure 9 that the economic development trend is relatively stable, but there are significant changes in 10∼20 iterations and 50∼60 iterations, mainly due to the changes in economic policies at that time. However, the accuracy of the overall evolution meets the demands.

### 4.5. Judgment Time of Prediction Results

The characteristic of intelligence is that the data has a large amount of data processing and high processing complexity, so the identification time of prediction results is another verification index. The results show that the identification time of prediction results in community public sports service capability *x*_*i*_, community public sports service status judgment *x*_*j*_, and public sports service trend judgment *x*_*k*_ is less than 40 seconds. Compared with 0∼10 iterations, the calculation time of 10∼20 iterations is longer, mainly due to the large amount of postprocessing data and the relatively complex calculation process. However, the identification time of the overall prediction results meets the requirements of the guidelines for the status of services in community public sports, and the results are shown in Table 3.

The overall calculation time of the level of public sports information can be derived from Table 3, as shown in Figure 10.

We can see in Figure 10 that the overall mounting time of the calculation result is better, between 0 and 1 s. That is, the overall mounting time is short. At the same time, under different iteration and accuracy requirements, the fitting time has not changed, indicating that the overall calculation time is relatively stable, which further proves the effectiveness of this method. Compared to the traditional simulated annealing algorithm, the computational time of the iterative simulated annealing algorithm is shorter.

## 5. Conclusion

The social economy is the basis for the development of community public sports. With the improvement of the economic level, the development of community public sports is getting better and better. The development and improvement of community public sports promotes the development of the social economy to a large extent and have an inseparable relationship. The rapid development of the intelligence level of the community public sports makes the intelligence level higher and higher (Tubishat [16]), and the data volume and complexity show characteristics (Twahirwa and Wang [17, 18]), which makes traditional analytical methods unable to meet the analytical requirements of relevant data institutions. The studies of Yagmur and Kesen [19] have resulted in a significant decline in the accuracy of forecast results. A method of analysis based on a simulation annealing algorithm is proposed in this document [20]. Through the standardized processing of public sports service data, fitting data with an accuracy of 0.1 is obtained (Svalina et al. [20]). Then, using iterative calculation, the prediction results and identification rates of public sports service capability judgment *x*_*i*_, public sports service status judgment *x*_*j*_, public sports service trend judgment *x*_*k,*_ and other indicators are obtained by Zolfi and Jouzdani [21, 22]. The MATLAB simulation results show that the recognition accuracy of the prediction results in the five indicators is >95% (Ilin [23]), while the initial threshold and the requirements in the guidelines for the development status of community public sports are 0.1. At the same time, the identification time of the prediction results in the five indicators is less than 7 seconds, and the identification time of the prediction results in the judgment of public sports service trend and intelligence level is less than 4 seconds (He and Ye [24]). So, the overall judgment result is better (Chen et al. [25]). The global adjustment time of the calculation result is better, between 0 and 1 s, i.e., the global adjustment time is short. At the same time, under different iteration and accuracy requirements, the fitting time has not changed, indicating that the overall calculation time is relatively stable, which further proves the effectiveness of this method. Compared with the classical simulated annealing algorithm, the calculation time of the iterative simulated annealing algorithm is shorter. However, there is still insufficient research on the coupling between public sports intelligence level indicators and intelligent judgment in this paper. In future research, we will focus on the analysis of the above contents.

## Figures and Tables

**Figure 1:** The data source of intelligent prediction of public sports in sports.

**Figure 2:** The demand for different sports for social public sports.

**Figure 3:** The correlation between community public sports and socioeconomic development.

**Figure 4:** Community public sports analysis steps.

**Figure 5:** Results of local and global adjustment.

**Figure 6:** The correlation between community public sport and social economy.

**Figure 7:** Accuracy of predictive results for each index.

**Figure 8:** Judgment on the service status of communal public sports.

**Figure 9:** Outcome of the judgment trend in public sports services.

**Figure 10:** The total fitting time.

**Table 1:** Degree of adjustment of the various figures.

The adequacy of predictive data on the level of public athletic information	Iteration (times)	Fitting degree (%)
Local fitting	0∼50	97.3
	50∼100	98.7

Global fitting	0∼50	97.2
	50∼100	99.6

Total fitting degree	0∼100	98.3

**Table 2:** Accuracy of forecast outcomes.

Judgment index	Iteration (times)	Fitting degree (%)
The community sports organizations	0∼50	98.23
	50∼100	97.23

The community members	0∼50	96.62
	50∼100	98.82

Venue facilities and funds	0∼50	97.02
	50∼100	98.32

Administrators	0∼50	97.12
	50∼100	98.24

The community sports activities	0∼50	97.22
	50∼100	97.12

Total fitting degree	0∼100	98.62

**Table 3:** Judgment time of forecast results.

Judgment index	Iteration (times)	Fitting degree (%)
The community sports organizations	0∼10	0.61 ± 1.23
	10∼20	0.53 ± 0.92

The community members	0∼10	0.32 ± 2.01
	10∼20	0.72 ± 2.32

Venue facilities and funds	0∼10	0.62 ± 1.72
	10∼20	0.72 ± 0.93

Administrators	0∼10	0.61 ± 1.91
	10∼20	0.73 ± 0.12

The community sports activities	0∼10	0.64 ± 1.84
	10∼20	0.71 ± 0.82

Total fitting time	0∼20	0.72 ± 2.01

## Data Availability

The data used to support the ﬁndings of this study are available from the corresponding author upon request.
